# Mesenchymal Stem/Stromal Cells as a Vehicle for Cytokine Delivery: An Emerging Approach for Tumor Immunotherapy

**DOI:** 10.3389/fmed.2021.721174

**Published:** 2021-08-27

**Authors:** Ehsan Razeghian, Ria Margiana, Supat Chupradit, Dmitry O. Bokov, Walid Kamal Abdelbasset, Faroogh Marofi, Siavash Shariatzadeh, Foad Tosan, Mostafa Jarahian

**Affiliations:** ^1^Human Genetics Division, Medical Biotechnology Department, National Institute of Genetics Engineering and Biotechnology (NIGEB), Tehran, Iran; ^2^Department of Anatomy, Faculty of Medicine, Universitas Indonesia, Jakarta, Indonesia; ^3^Cipto Mangunkusumo Hospital, The National Referral Hospital, Central Jakarta, Indonesia; ^4^Master's Programme Biomedical Sciences, Faculty of Medicine, Universitas Indonesia, Jakarta, Indonesia; ^5^Department of Occupational Therapy, Faculty of Associated Medical Sciences, Chiang Mai University, Chiang Mai, Thailand; ^6^Institute of Pharmacy, Sechenov First Moscow State Medical University, Moscow, Russia; ^7^Laboratory of Food Chemistry, Federal Research Center of Nutrition, Biotechnology and Food Safety, Moscow, Russia; ^8^Department of Health and Rehabilitation Sciences, College of Applied Medical Sciences, Prince Sattam bin Abdulaziz University, Al Kharj, Saudi Arabia; ^9^Department of Physical Therapy, Kasr Al-Aini Hospital, Cairo University, Giza, Egypt; ^10^Immunology Research Center (IRC), Tabriz University of Medical Sciences, Tabriz, Iran; ^11^Department of Pharmacology, School of Medicine, Shahid Beheshti University of Medical Sciences, Tehran, Iran; ^12^Student Research Committee, Semnan University of Medical Sciences, Semnan, Iran; ^13^Toxicology and Chemotherapy Unit (G401), German Cancer Research Center, Heidelberg, Germany

**Keywords:** mesenchymal stem/stromal cells, cytokine, tumor-immunotherapy, gene therapy, cytokine delivery

## Abstract

Pro-inflammatory cytokines can effectively be used for tumor immunotherapy, affecting every step of the tumor immunity cycle. Thereby, they can restore antigen priming, improve the effector immune cell frequencies in the tumor microenvironment (TME), and eventually strengthen their cytolytic function. A renewed interest in the anticancer competencies of cytokines has resulted in a substantial promotion in the number of trials to address the safety and efficacy of cytokine-based therapeutic options. However, low response rate along with the high toxicity associated with high-dose cytokine for reaching desired therapeutic outcomes negatively affect their clinical utility. Recently, mesenchymal stem/stromal cells (MSCs) due to their pronounced tropism to tumors and also lower immunogenicity have become a promising vehicle for cytokine delivery for human malignancies. MSC-based delivery of the cytokine can lead to the more effective immune cell-induced antitumor response and provide sustained release of target cytokines, as widely evidenced in a myriad of xenograft models. In the current review, we offer a summary of the novel trends in cytokine immunotherapy using MSCs as a potent and encouraging carrier for antitumor cytokines, focusing on the last two decades' animal reports.

## Introduction

Cytokines as a family of molecular messengers support the communications between immune cells to establish a harmonized, strong, while self-limited reaction to a target antigen (1–3). Although a diversity of the correlation of the immune system befalls by direct cell-cell contact, the release of cytokines provides the robust and swift spreading of the immune signaling axis in a multifaceted and well-organized mode (4–6). The rising proofs over the last two decades in harnessing the immune system to eliminate tumor cells have been sustained by reinforced efforts for characterizing and utilizing the massive signaling networks of cytokines for advancing tumor therapy (7, 8).

Cytokines typically induce both immune effector cells and also stromal cells at the tumor area and improve transformed cell recognition through cytotoxic effector cells (9–11). Frequent *in vivo* reports have shown that a diversity of cytokines, ranging from interleukins (ILs) to interferons (IFNs), and also tumor necrosis factor-related apoptosis-inducing ligand (TRAIL), have unique antitumor competencies, highlighting the importance of their application for cancer therapy (12–14). Nonetheless, the wide-ranging pleiotropism and redundancy of cytokine axis concomitant with the dual activity of various cytokines in both immune induction and immune inhibition, and also treatment-related toxicities, poses substantial controversies to our aptitude for achieving expressive antitumor outcome (8, 15). For instance, some evidence is implying that the low response rate and high toxicity correlated with high-dose IL-2 and IFN-α therapy could disturb their clinical use (8).

Presently, mesenchymal stem/stromal cells (MSCs), a well-known multipotent stromal cell, have been employed as a carrier for gene and drug delivery (16, 17). Remarkably, MSC utility is a capable strategy for the progress of gene therapy and drug-loading approaches due to their intrinsic attributes, importantly remarkable homing capacity, and tumor tropism (18). Also, another unique property of MSC is its lower immunogenicity due to the minimized expression of costimulatory molecules (19, 20), thus signifying that there is no need for the application of immunosuppressive drugs before allogeneic transplantation. These properties introduce them as an encouraging option for cellular-based immunotherapy as a drug or cytokine delivery vehicle (21–23). Correspondingly, through the combining inherent cell characteristics and antitumor activities of cytokines, the use of MSCs engineered to express target cytokines offers more competent cytokine delivery to tumor tissue and thereby seems to be a rational and promising approach in the context of tumor immune therapy (Figure 1). For example, it was found that intratumoral infusion of MSCs modified to overexpress IL-12 (MSC-IL-12) could result in the more prominent tumor-specific T-cell responses and antitumor impacts, and also more continued expressions of IL-12 and IFN-γ in both sera and tumor tissues than the injection of IL-12-expressing adenovirus (rAd/IL-12) in tumor-bearing xenografts (24). In addition, MSC-based delivery of TRAIL could make dramatically susceptible TRAIL-resistant tumor cells to TRAIL-induced apoptosis in xenografts (25).

**Figure 1:** Mesenchymal stem/stromal cell (MSC)-based cytokine delivery for tumor immunotherapy. Human MSCs upon procurement from various sources, such as bone marrow (BM), adipose tissue, and umbilical cord (UC), can be modified to express therapeutic genes (e.g., cytokines) for exerting antitumor response in patients suffering from tumors.

Herein, we will discuss recent findings respecting the antitumor effects of cytokine delivery using MSCs, with a special focus on the last two decades of *in vivo* studies.

## Cytokine-Based Tumor Immunotherapy

Cytokines are polypeptides or glycoproteins with molecular weight ranging from typically 6 to 70 kD and largely support proliferation, activation, differentiation, and inflammatory or anti-inflammatory signals to diverse cell types (26–28). They are commonly produced throughout a well-defined duration in response to a stimulus, and also display short-lived autocrine or paracrine effects because of their restricted half-life in the circulation (8, 29). Nonetheless, IL-7 or hematopoietic growth factors are secreted homeostatically in an incessant style (8). Upon the detection of the effective antitumor functions of various pro-inflammatory cytokines in preclinical models, comprehensive clinical studies have resulted in the approval of recombinant IFN-α and IL-2 to treat various malignancies usually with modest effectiveness. These primary landmarks in tumor immunotherapy have been followed by advanced immune checkpoint inhibitors (30–32) and also chimeric antigen receptor (CAR)-T cells (33–35). A renewed attention to the anticancer attributes of cytokines has sustained a pronounced increase in the number of clinical trials for addressing the safety and efficacy of cytokine-based components either as single agents or in combination with other immunomodulatory ingredients (Table 1). Indeed, cytokines hinder tumor cell development primarily by antiproliferative or proapoptotic functions, and secondarily through eliciting the cytotoxic effects of immune cells toward tumor cells. In the 1970s, Gresser and Bourali (36) for the first time described the antitumor property of IFN-α vs. tumor cell line-bearing mice. In the 1980s and 1990s, this finding was followed by the progress of recombinant DNA technologies, causing many preclinical and clinical studies of the possible antitumor effects of some recombinant cytokines. However, their short half-life and narrow therapeutic windows, and modest antitumor effectiveness obstruct their utility in the clinic. To date, only IL-2 and IFN-α have displayed mild clinical efficacy, and thereby have received the approval of the Food and Drug Administration (FDA) for various malignant disease therapy. The IL-2 has been approved for advanced renal cell carcinoma (RCC) therapy (37) and metastatic melanoma (38), while IFN-α has been approved for the treatment of hairy cell leukemia (HCL) (39), non-Hodgkin lymphoma (NHL) (40), melanoma (41), and AIDS-related Kaposi's sarcoma (42). Nevertheless, in addition to the listed challenges and controversies, high toxicity and neurological side effects related to high-dose IL-2 and IFN-α therapy mainly due to the pleiotropic effect of cytokines is another factor limiting their extensive application (43). For instance, Kruit et al. found that a high-dose regimen of IL-2 and IFN-α therapy in combination with lymphokine-activated killer cells caused three treatment-associated deaths in patients suffering from metastatic RCC. Furthermore, hypotension, cardiotoxicity, pulmonary edema, renal toxicity, and infectious complications were observed following intervention (44). Moreover, the high-dose IFN-α therapy (HDI) led to constitutional symptoms, chronic fatigue, myelosuppression, elevated liver enzyme levels, and neurologic symptoms in patients with high-risk melanoma (45). Thereby, finding novel strategies to overcome high toxicities, short half-life, and pleiotropic effects of cytokines is of paramount importance.

**Table 1:** Completed clinical trials (phases 3 and 4) respecting cytokine-based immunotherapy for treatment of human cancers registered in ClinicalTrials.gov (May 2021).

**Condition**	**Cytokine**	**Phase**	**Participant number**	**Location**	**NCT number**
Kidney cancer	IL-2	3	NA	USA	NCT00018941
Kidney cancer	IL-2	3	220	France	NCT00416871
Colon cancer	IFN-α	3	796	Germany	NCT01060501
Kidney cancer	IL-2	3	96	UK	NCT00053807
	IFN-α				
Kidney cancer	IL-2	4	NA	USA	NCT00006864
Lymphoma	IL-2	3	206	USA	NCT00002649
Leukemia	IFN-α	3	744	USA/UK	NCT00002868
Leukemia	IFN-α	4	360	Spain	NCT00390897
Leukemia	IFN-α	3	1551	Germany/Switzerland	NCT00055874
Colon cancer	IFN-α	3	598	Austria	Completed
Multiple myeloma	IFN-α	3	103	Italy	NCT00633542
Multiple myeloma	IFN-α	3	244	NA	NCT00732641
Multiple myeloma	IFN-α	2/3	350	Austria	NCT00205751
Kidney cancer	IL-2	3	670	Multinational	NCT00053820
	IFN-α				
Kidney cancer	IL-2	3	69	USA	NCT00003126
Kidney cancer	IFN-α	3	NA	Multinational	NCT00005966
Kidney cancer	IFN-α	3	320	Multinational	NCT00005966
Kidney cancer	IL-2	3	456	France	NCT00416429
	IFN-α				
Kidney cancer	IFN-α	3	732	USA/Canada	NCT00072046
Bladder cancer	IFN-α	2/3	140	Singapore	NCT00330707
Melanoma	IL-2	3	140	USA	NCT00002882
	IFN-α				
Various cancers	IL-11	3	62	China	NCT01663441
Melanoma	IL-2	3	70	France	NCT00200577
Melanoma	IL-2	3	350	Multinational	NCT00039000
Melanoma	IFN-α	3	269	Italy	NCT01359956
Melanoma	IFN-α	3	3000	USA	NCT00004196
Melanoma	IFN-α	3	901	Germany	NCT00204529
Liver cancer	IFN-α	4	100	Japan	NCT00375661
Kidney cancer	IL-2	3	310	Italy	NCT00502034
	IFN-α				
Leukemia	IL-2	3	360	Multinational	NCT00003991
Leukemia	IL-2	3	420	France	NCT00931138
Leukemia	IL-2	3	61	USA	NCT00002945
Leukemia	IL-2	4	84	Sweden	NCT01347996
Leukemia	IL-2	3	720	USA	NCT00006363
Kidney cancer	IFN-α	3	626	Multinational	NCT00065468
Head and neck cancer	IFN-α	3	NA	Multinational	NCT00054561
Kidney cancer	IFN-α	3	649	Multinational	NCT00738530
Melanoma	IFN-γ	3	122	USA	NCT00001296
Liver cancer	IFN-α	4	120	Taiwan	NCT00630084
Liver cancer	IFN-α	3	150	Italy	NCT00273247
Multiple myeloma	IFN-α	3	312	USA	NCT00002556
Melanoma	IFN-α	3	167	USA	NCT00003444
Leukemia	IFN-α	3	1106	Multinational	NCT00333840
Leukemia	IFN-α	3	96	USA	NCT00050531
Leukemia	IFN-α	3	41	Germany	NCT02736721

## MSC Tropism Into the Tumor

Human MSCs have demonstrated possible clinical utility for tumor therapy because of their inherent tumor tropism, making them promising carriers for antitumor drugs or molecules (17, 46–48). Previous evaluations of MSC function in recipients have been carried out based on the visual observations in host tissue upon the sacrifice, and thereby impedes tracking of MSC *in vivo* (49). However, various approaches such as *in vivo* bioluminescent (BLI) imaging have currently provided the possibilities to elucidate circumstances in which MSC specifically engraft in the target area (e.g., injured tissue or tumor site). For instance, Kidd et al. found that intravenously injected engineered MSCs to express firefly luciferase (ffLuc-MSC) experienced persistent and selective colocalization with tumor tissue in syngeneic and xenogeneic breast tumor-bearing murine, as shown by bioluminescent detection of administered MSCs (18). A similar pattern of tumor tropism was also observed in the ovarian tumor model upon intraperitoneal injection of modified MSC (18). Remarkably, these findings have indicated that MSC tumor tropism is independent of tumor type, immunocompetence, and also administration route (18). Monitoring of the migration and incorporation of magnetically labeled MSCs using magnetic resonance (MR) imaging evidenced that MSCs could show efficient migration toward glioma tissue in glioma cell-bearing Fischer 344 rats with high specificity in a temporal-spatial pattern (50). Meanwhile, co-labeled MSCs with superparamagnetic iron oxide nanoparticles (SPIO) and enhanced green fluorescent protein (EGFP) were detectable at the border between the tumor and normal parenchyma for 2 weeks post-transplantation (50). Also, it has been suggested that the administration of ionizing radiation (IR) to glioma tumors might restore MSC tropism to tumor tissue (51). Correspondingly, IR considerably improved the tropism of MSCs to patient-derived glioma stem-like GSC7-2 cell-bearing murine. Immunohistochemistry analysis indicated an improved CCL2 in irradiated GSC7-2 gliomas, suggesting that chemokine CCL2 was reliable for IR-stimulated tropism of MSCs to tumor tissue (51). Also, MSC tropism to tumor tissue could be ameliorated by valproic acid (VPA) (52), and also promotion of the expression of the activated lymphocyte cell adhesion molecule (ALCAM) and N-cadherin mediated by downregulation of microRNA-192 and microRNA-218 *in vivo* (53). Furthermore, investigation of the interrelation between adipose tissue-derived MSCs (ADSCs) and MCF-7 breast cancer cells in a Matrigel coculture condition as well as in a nude mouse model supported the hypothesis that MCF-7 improved the tumor tropism of ADSC, which was adjusted by chemokines, including the macrophage inflammatory protein (MIP)-1δ and MIP-3α (54). Also, ADSCs showed tropism and triggered tumorsphere creation of MCF-7 cells (54). Besides, there is an indication showing that MSCs could infiltrate the tumor tissue in osteosarcoma xenografts (55). However, MSCs seem to be eliminated by splenic macrophage phagocytosis and therefore restrained the more efficient tumor engraftment (55). Nonetheless, transiently exhausted macrophages with liposomal clodronate, a potent antimacrophage agent, may lead to improved MSC localization within a tumor without marked diminishment in tumor-associated macrophages (TAMs), providing a novel strategy for the restoration of the clinical efficacy of MSCs as a carrier for antitumor agents (55).

## MSCs as a Carrier for ILs

### MSCs as a Carrier for IL-2

The IL-2 largely contributes to the stimulation of the immune system which could result in cancer elimination. As described, IL-2 has been shown capable of arbitrating tumor deterioration and was verified for metastatic renal cell carcinoma and metastatic melanoma by the FDA (56). Recent studies have shown that IL-2 gene-engineered MSCs (MSC-IL-2) could be considered a rational strategy for treating human tumors as IL-2 antitumor function accompanied with MSC efficient tropism. For instance, in addition to the migratory competence of MSCs *in vivo*, intratumoral injection of MSC-IL-2 led to the robust regression of glioma tumor growth and also improved overall survival rate of 9L glioma cell-bearing rats (57). However, the study of the possible effects of ADSCs modified to express IL-2 on B16F10 melanoma cell xenografts revealed that systemic injection of the modified MSCs also could effectively engraft into melanoma lung tumors but could not affect melanoma pulmonary metastases, and also the survival rate of the animal (58). In another study, hADSC-IL-2 potently induced activation of peripheral blood mononuclear cells (PBMCs) and conversely reduced proliferation and survival of SH-SY5Y neuroblastoma cells *in vitro*. However, a conditioned medium from hADSC-IL2 supported the proliferation of SH-SY5Y cells despite the activation of T cells, natural killer (NK) cells, NKT cells, and activated T killers, suggesting therapies using this cytokine have to be taken into careful consideration (59). On the other hand, cytochalasin-B, a cell-permeable mycotoxin-induced human ADSC-IL-2-derived extracellular vesicle (EV) could stimulate more effective CD8+ T killers than ADSC-IL-2 to eliminate human triple-negative breast cancer MDA-MB-231 and MDA-MB-436 cells *in vitro* (60).

### MSCs as a Carrier for IL-12

IL-12 has been found to adjust NK cells and cytotoxic T-lymphocyte (CTL) immunities in tumor therapy. A well-known function of IL-12 is its aptitude to stimulate IFN-γ secretion from NK cells, and also CD4+ and CD8+ T cells (61).

Gene therapy in Ewing sarcoma using MSCs as a carrier for IL-12 could suppress tumor development. Accordingly, IL-12 expression was detected in tumor tissue in TC71 Ewing sarcoma xenografts following systemic injection of MSC-IL-12, leading to the suppressed tumor growth compared with control xenografts (62). Similarly, genetically modified MSCs by lentivirus-mediated mouse IL-12 could modify malignant ascites in murine (63). In addition to the critical chemotactic effects on dendritic cells (DCs) *in vitro*, and also pronounced safety *in vivo*, MSC-IL-12 robustly attenuated not only the volume of ascites but also red blood cell (RBC) frequency in ascites, ultimately facilitating promoted survival period of the experimental model (63). Besides, MSC-IL-12 intratumoral injection resulted in abrogated tumor progress in established subcutaneous B16BL6 tumors; however, the intravenous administration of MSC-IL-12 did not hinder the tumor development in melanoma B16BL6 cell-bearing animals (64). These findings delivered the proof of the concept that MSCs are largely distributed in the lungs, and therefore their administration by intravenous route could not possibly mitigate the development of the human solid tumors (64). Other studies showed that human umbilical cord mesenchymal stem/stromal cells infected by an adenoviral vector encoding IL-12 (UC-MSC-IL-12) could negatively modify tumor development in breast carcinoma SKOV3 cell xenografts (65). In the tumor-bearing nude mice model, the systemic administration of MSCs led to a noticeable regression in the development of SKOV3 tumor explants. Also, MSC-IL-12-derived conditioned medium (CM) suppressed the proliferation of SKOV3 cells and stimulated cell death *in vitro* (65). In another study, injection of MSC-IL-12 into Ast11.9-2 glioma cell-bearing C57/B16 mice caused enhanced NK cell infiltration in brain tissue, and thereby exerted an improvement in non-specific cell lysis, while could not induce significant promotion in overall survival rates of the treated mice compared with control mice (66). Nonetheless, it was demonstrated that treatment with Fuzheng Yiliu decoction (FYD), a traditional Chinese medicine, in combination with MSC-IL-12 therapy could elicit synergistic antitumor effects in glioma-bearing nude mice (67). Meanwhile, glioma U251 cell-bearing BALB/c nude mice experienced robust decreases in tumor volume upon treatment with FYD plus MSC-IL-12. Moreover, a combine treatment of FYD and MSC-IL-12 induced higher Bax and lower Bcl-2 expression and also supported higher serum IL-12 and INF-γ levels compared with monotherapy with FYD or MSC-IL-12 (67). Besides, intramural injection of genetically modified MSCs co-expressing IL-12 and IL-7 caused a marked inversion of the CD4+/CD8+ T-cell ratio with an intricate antitumor response mainly mediated by CD8+ effector T cells in glioma tumor-bearing mice (68). Furthermore, MSCs constitutively secreting IL-12 were able to exert a potent regression in the growth of renal cell carcinoma (RCC), and thereby improved the survival rate of the tumor-bearing mice predominantly through the induction of NK cell activation and IFN-γ secretion (69).

### MSCs as a Carrier for IL-18

The IL-18 was first recognized as a potent IFN-γ-inducing molecule. This cytokine induces IFN-γ secretion from NK cells and T-helper-type 1 cells, in particular, in a marked synergy with the greatly strong and toxic cytokine IL-12 (70).

Current studies have exhibited that hUMSCs modified to overexpress IL-18, but not parental hUMSCs, could counteract proliferation, migration, and invasion of breast tumor MCF-7 (71) and HCC1937 cells (72) *in vitro*. Analyses have indicated that stimulation of G1- to S-phase arrest of tumor cells was reliable for the hUMSC-IL-18-mediated suppressive effects on the proliferation of these cells (72). More importantly, hUMSC-IL-18 injection to breast cancer 4T1 cell-bearing BALB/c mice supported noticeable abrogation in tumor cell growth *in vivo* by activating immunocytes and immune cytokines, and also constraining tumor angiogenesis, as evidenced by reduced CD31 expression in hUMSC-IL-18 group compared with the control group (73). Likewise, intratumoral injection of MSC-IL-18 into glioma C6 cell-bearing Sprague-Dawley rats elicited delayed tumor growth of glioma, and thereby provided extended survival in experimental models (74). The existence of the association between the transplantation of MSCs constitutively secreting IL-18 and ameliorated T-cell infiltration and continued antitumor responses have indicated that IL-18 can be an operative and rationally adoptive immunotherapy for malignant tumors (74).

### MSCs as a Carrier for IL-21

The IL-21 as a pro-inflammatory cytokine has been advanced as an immunotherapeutic option because of its potent influences on NK cells and T cells; however, the clinical achievement in tumor patients has been restricted (75).

It has been currently supposed that MSCs genetically modified to express IL-21 (MSC-IL-21) could improve antitumor activities through localized delivery of IL-21. For instance, MSC-IL-21 systemic injection into the B-cell lymphoma A20 cell-bearing BALB/c mice resulted in delayed tumor occurrence and also prolonged survival, while either MSCs or recombinant adenovirus-expressing IL-21 (rAD/IL-21) could not induce desirable antitumor effects in experimental models (76). Respecting the observations, the evident antitumor impacts were mediated by the pronounced levels of IL-21 delivered to the liver, averting the establishment of a tumor nodule. Remarkably, MSC-IL-21 therapy caused stimulation of effector T and NK cells but strongly hindered the activities of immune suppressor cells (76). Moreover, hUC-MSC-IL-21 suggestively weakened SKOV3 (77) and A2780 (78) ovarian cancer volume in xenografts by affecting the serum levels of IFN-γ and TNF-α, concurrently restoring the expression of natural killer group 2 member D (NKG2D) and MHC class I polypeptide-related sequence A (MICA) molecules in the tumor microenvironment (77). Also, abrogation of SKOV3 ovarian cancer growth in mice may arise from negative regulation of β-catenin and cyclin-D1 in the TME (77).

Moreover, combine treatment of hUCMSC-IL-21 and miR-200c supported more prominent antitumor effects than monotherapy with hUCMSC-IL-21on SKOV3 cell-bearing mice mainly through boosting the serum levels of IFN-γ, IL-21, and TNF-α and also the splenocyte cytotoxicity (79). Also, the expression of β-catenin, cyclin-D1, Gli1, Gli2, and Zinc finger E-box-binding homeobox 1 (ZEB1) was reduced, and conversely, the expression of E-cadherin, a downstream target of miR-200c, was improved in tumor tissues of murine treated with hUCMSC-IL-21 plus miR-200c (79). These findings emphasize the significance of the repression of Wnt/β-catenin signaling and inhibiting the epithelial-mesenchymal transition (EMT) to attain the favorite outcome in patients suffering from the ovarian tumor (79). A potent decrease in proliferation and migration in reproductive cancer cells transfected with miR-200c mimic implies miR-200c prominence to be utilized as a possible antitumor molecule (80).

A summary of preclinical studies respecting IL delivery using MSCs is listed in Table 2.

**Table 2:** The overview of studies based on the use of mesenchymal stem/stromal cells (MSCs) as a carrier for delivery of interleukins to treat human tumors (*in vitro* and *in vivo*).

**Cancer**	**Interleukin**	**Cell line/model**	**Results (Ref)**
Glioma	IL-2	9L glioma cell line	Inhibition of the proliferation of 9L cell *in vitro* (57)
		9L glioma cell-bearing rats	MSC-IL-2 efficient tropism into tumor area and reducing tumor burden (57)
Neuroblastoma	IL-2	SH-SY5Y neuroblastoma cell line	Reducing the SH-SY5Y proliferation and also activation of PBMCs *in vitro* (59)
Breast cancer	IL-2	MDA-MB-231 cell line	Induction of apoptosis in MDA-MB-231 cells (60)
Melanoma	IL-2	B16F10 melanoma cell line	Increasing the viability and reducing the apoptosis of melanoma cells *in vitro* (an unexpected result) (58)
		B16F10 cell-bearing mice	Reducing the systemic CD4+ cells without any effect on tumor size in melanoma bearing mice (58)
Ascites	IL-12	MethA ascites mice models	Suppression of the growth of ascites and promotion of the survival of tumor-bearing mice (63)
Melanoma	IL-12	B16F10 cell-bearing mice	Attenuation of tumor burden by MSC-IL-12 intratumoral but not an intravenous injection (64)
Ovarian cancer	IL-12	SKOV3 cell line	Inhibition of the proliferation of SKOV3 cells and inducing the cellular apoptosis *in vitro* (65)
		SKOV3 cell-bearing nude mice	Suppression of the development of SKOV3 tumor explants (65)
Glioma	IL-12	U251 cell-bearing nude mice	Inducing the marked inhibitory effect toward tumor growth by improvement of Bax/Bcl-2 ratio leading to tumor cells apoptosis (66)
Renal carcinoma	IL-12	786-0 cell-bearing nude mice	Regression tumor growth and providing prolonged mice survival (69)
Glioblastoma	IL-12	GL261 and CT2A cell-bearing mice	Remarkable inversion of the CD4+/CD8+ T-cell ratio and inducing the CD8+ effector T-cell-mediated antitumor response (68)
	IL-7		
Breast cancer	IL-18	MCF-7 cell line	Inhibition of the proliferation, migration, and invasion of the MCF-7 cell *in vitro* (71)
		MCF-7 cell-bearing mice	Suppression of the proliferation and metastasis of breast tumor cell *in vivo* (71)
Glioma	IL-18	Glioma C6 cell line	Suppression of the growth of C6 cells *in vitro* (74)
		C6 glioma-bearing SD rats	Inhibition of the growth of glioma cell leading to prolonged survival (74)
Lymphoma	IL-21	A20 cell-bearing BALB/c mice	Supporting the inhibited tumor incidence as well as promoted survival (76)
Ovarian cancer	IL-21	SKOV3 cell-bearing nude mice	Suppression of the β-catenin and cyclin-D1 activities in the tumor tissues leading to delayed tumor growth *in vivo* (77)
Ovarian cancer	IL-21	A2780 cell-bearing nude mice	Delayed tumor growth by activation of NK cells response against tumor cells *in vivo* (78)
Ovarian cancer	IL-21	SKOV3 cell-bearing nude mice	Inhibition of tumor growth by combination therapy using MSC-IL-21 and miR-200 mediated by inhibition of the Wnt/β-catenin signaling axis and also epithelial-mesenchymal transition (EMT) *in vivo* (79)

*IL, interleukin; PBMC, peripheral blood mononuclear cell*.

## MSCs as a Carrier For IFNs

### MSCs as a Carrier for IFN-α

IFN-α is a pleiotropic cytokine, which can widely be employed for the therapy of patients with tumors and viral disease (81). In addition to affecting multiple biologic processes of tumor cell, it can support both differentiation and activities of host immune cells. Preclinical reports in mouse tumor models show the significance of host immune mechanisms in the exerting prolonged antitumor functions following the treatment of an animal with IFN-α and IFN-β (82); however, IFN-α may cause some untoward effects because of its short half-life and high dose (81).

Investigation of the clinical effects of hepatocellular carcinoma (HCC) treatment with human bone marrow (BM)-MSCs modified to overexpress IFN-α2b indicated the intervention caused delayed tumor growth in HepG2 cell-bearing NOD/SCID mouse through the negative regulation of the Notch signaling axis. Moreover, CM derived from modified MSCs induced G2/M phase arrest in HepG2 and Huh7 cells *in vitro* (81). Similarly, systemic injection of the BMMSC secreting IFN-α abridged the development of B16F10 melanoma cells and substantially extended survival in C57BL/6 mice with melanoma. Analysis signified robust elevation in apoptosis and a reduction in proliferation and blood vasculature in tumor tissue (83). Likewise, subcutaneous injection of BMMSC-IFN-α modified the tumor growth *in vivo* and sustained the overall survival in mice multiple myeloma model (84). It was found that observed antitumor effects were dependent on the promoted apoptosis of tumor cells, a decrease in microvessel density, and ischemic necrosis (84). Nonetheless, systemic injection of BMMSC-IFN-α had no significant effect on the survival of mice largely because of the substantial entrapment of administered cells in the pulmonary vessels and thereby suggests the superiority of intratumoral injection of modified cells over systemic injection in terms of clinical efficacy in preclinical models (84).

### MSCs as a Carrier for IFN-β

Recent finishings have shown that IFN-β gene delivery could stimulate apoptosis in IFN-β-resistant cancer cells, such as, melanoma, glioma, and renal cell carcinoma (RCC) (85). It has been found that the genetically modified MSCs to generate IFN-β could induce apoptosis in prostate cancer cell line PC-3 *in vitro*. Also, systemic injection of these modified MSCs could lead to the diminished proliferation of transformed cells in both PC-3 (86) and TRAMP-C2 (87) xenografts, as documented by reduced tumor weight, leading to the prolonged animal survival (86). Furthermore, IFN-β-secreting BMMSCs (BMMSC-IFN-β) in addition to the induction of reduced cell proliferation and G1-phase arrest in HCC cell line HepG2 and Huh7 *in vitro*, suppressed tumor growth in HCC NOD/SCID mice model. Molecular analysis indicated that downregulation of the AKT/Forkhead box O3 (FOXO3a) pathway plays a central role in observed antitumor effects in xenografts (88). Also, systemic injection of the MSC-IFN-β resulted in high levels of IFN-β secreted by MSC in the tumor microenvironment but not in circulation in breast cancer 4T1 cell-bearing mice. Furthermore, intervention supported inhibition of the signal transducer and activator of transcription 3 (STAT3) signaling axis and also dramatically decreased pulmonary and hepatic metastases in xenografts (89). Besides, canine ADMSC-IFN-β co-cultured with canine melanoma LMeC cells led to the pronounced cell cycle arrest in tumor cells and significantly diminished cyclin D1 expression in these cells. Regardless of the affecting proliferation of LMeC cell, ADMSC-IFN-β induced active forms of caspase-3 and Bak in co-cultured LMeC cells, and thereby elicited their apoptosis *in vitro* (90). Remarkably, intratumoral injection of canine ADMSC-IFN-β plus cisplatin into melanoma B16F10 cells bearing C57BL/6 mice resulted in the more prominent antitumor effects than monotherapy with ADMSC-IFN-β and cisplatin (91). These findings confirmed the possible capability of ADMSC-mediated IFN-β for the treatment of canine and human cancer patients (91). Additionally, IFN-β producing human UC-MSCs could induce robust apoptosis in human triple-negative breast (TNBC) carcinoma cell lines MDA-MB-231 and Hs578T *in vitro* (92), and in bronchioloalveolar carcinoma xenografts in SCID mice *in vivo* (93). Furthermore, administration of the IFN-β-secreting human MSCs into tongue squamous cell carcinoma (TSCC) (94), and also glioma xenografts (95) exerted dramatic antitumor responses *in vivo*.

### MSCs as a Carrier for IFN-γ

The IFN-γ while stimulates the expression of resistant genes in tumor cells, this signaling sponsored the maturation of NK and innate lymphatic cells (ILCs), and also the generation of CXCL9 and CXCL10 in immune cells for improving T-cell infiltration (96).

It has been displayed that MSCs engineered to deliver IFN-γ could eliminate tumor cells by continued activation of the TRAIL pathway, a potent stimulator of apoptosis. Meanwhile, IFN-γ-secreting MSCs stimulated apoptosis in lung tumor H460 cells mediated by TRAIL signaling pathways and resultant caspase-3 activation *in vitro*. Also, IFN-γ-modified administration of MSCs caused suppressed tumor growth in lung carcinoma xenografts (97). Furthermore, Tsujimura et al. found that murine MSC line C3H10T1/2 engineered to coexpress IFN-γ and herpes simplex virus-thymidine kinase (HSV-TK) in combination with prodrug ganciclovir could dramatically inhibit the proliferation of murine adenocarcinoma colon26 cell in xenografts (98).

A summary of preclinical studies respecting IFN delivery using MSCs is listed in Table 3.

**Table 3:** The overview of studies based on the use of mesenchymal stem/stromal cells (MSCs) as a carrier for delivery of interferons to treat human tumors (*in vitro* and *in vivo*).

**Cancer**	**Interferon**	**Cell line/model**	**Results (Ref)**
Liver cancer	IFN-α	HepG2 and Huh7 cell line	Inhibition of the proliferation and induction of G2/M phase arrest in HepG2 and Huh7 cell line by down-regulation of Notch signaling axis (81)
		HCC tumor-bearing SCID mice	Inhibition of tumor growth in SCID mice (81)
Melanoma	IFN-α	B16F10 cell-bearing C57BL/6 mice	Attenuation of the growth of B16F10 melanoma cells, and thereby inhibition of lung metastasis in melanoma leading to the prolonged survival (83)
Plasmacytoma	IFN-α	Sp6 cell-bearing BALB/c mice	Induction of apoptosis of tumor cells, reduction in microvessel density, and ischemic necrosis in tumor-bearing mice (84)
Prostate cancer	IFN-β	PC-3 cell line	Inhibition of the proliferation of PC-3 cells *in vitro* (86)
		PC-3 cell-bearing mice	Attenuation of PC-3 xenograft tumor weight and enhancing the mice survival (86)
		TRAMP-C2 cell-bearing mice	Marked attenuation in tumor volume (87)
Liver cancer	IFN-β	HepG2 and Huh7 cell line	Inhibition of the proliferation and induction of G1 phase arrest in HepG2 and Huh7 cell line by downregulation of AKT/FOXO3a pathway (88)
		HCC -bearing NOD/SCID mice	Suppression of HCC growth *in vivo* (88)
Squamous cell carcinoma	IFN-β	CAL27 cell line	Suppression of the proliferation of CAL27 cells *in vitro* and *in vivo* (94)
		CAL27 cell-bearing BALB/c mice	
Breast cancer	IFN-β	4 T1 cell-bearing mice	Inhibition tumor growth by inhibition of STAT3 signaling resulted in diminished pulmonary and hepatic metastases (89)
Melanoma	IFN-β	LMeC cell line (canine)	Induction of tumor cell apoptosis by up-regulation of caspase-3 and Bak (90)
Melanoma	IFN-β	B16F10 cell-bearing C57BL/6 mice	Inhibition of the growth of melanoma leading to the prolonged survival by combine treatment of MSC-IFN-β and cisplatin (91)
Glioma	IFN-β	F98 cell-bearing rat	Hindrance of glioma growth by marked Batf3+ dendritic cells and CD8+ T-lymphocyte infiltration into tumor tissue (99)
Glioma	IFN-β	9L glioma cell-bearing rat	Induction of tumor cell apoptosis, promotion of the antitumor cytokine secretion and CD4+ and CD8+ T-cell recruitment in intracranial glioma tissues (100)
	Il-18		
Breast cancer	IFN-β	MDA-MB-231 cell line	Obstruction of the tumor growth through apoptosis (92)
Bronchioloalveolar carcinoma	IFN-β	H358 cell line	Inducing H358 cell apoptosis *in vitro* (93)
		H358 cell-bearing SCID mice	Delayed tumor growth by stimulating apoptosis *in vivo* (93)
Bladder cancer	IFN-β	T24M cell-bearing mice	Pronounced suppression of tumor growth leading to the prolonged survival of mice (101)
Lung cancer	IFN-γ	H460 cell-bearing nude mice	Suppression of the growth and progression of lung carcinoma by caspase-3 activation (97)
Colon cancer	IFN-γ	colon26 cell-bearing nude mice	Inhibition of the proliferation of murine colon26 cell *in vivo* (98)

*IFN, interferon; FOXO3a, Forkhead box O3; HCC, hepatocellular carcinoma; STAT3, signal transducer and activator of transcription 3*.

## MSCs as a Carrier for Trail

The immune cytokine TRAIL has attracted substantial attention as an antitumor agent because of its competence to selectively induce tumor cell apoptosis without exerting toxicity *in vivo*. Nonetheless, poor circulation half-life, inadequate delivery to target cells, and TRAIL resistance have obstructed clinical translation (102).

### The Mechanism of Resistance to Cytokine TRAIL

TRAIL interrelates with two agonistic receptors, involving TRAIL-R1 (DR4) and TRAIL-R2 (DR5), and three antagonistic receptors, including TRAIL-R3 (DcR1), TRAIL-R4 (DcR2), and soluble receptor osteoprotegerin (OPG) (103, 104). Correspondingly, induction of either extrinsic or intrinsic apoptosis pathways in tumor cells resulting from binding of TRAIL to DR4 and DR4 is mainly induced by trimerization of responding receptors and establishment of the death-inducing signaling complex (DISC) (105, 106). Fas-associated death domain protein (FADD) is then engaged to the DISC and connects with the death domains (DD) located in the cytoplasmic domain of DR4 and DR5. Finally, this interaction supports translocation and subsequent stimulation of procaspase-8/10 (107).

Concisely, upregulation of antiapoptotic proteins, such as Bcl-2, c-FLIP, Mcl-1, and survivin, and also overactivation of survival or proliferation-involved signaling axis (e.g., NF-κB, PI3K/AKT, and ERK) play a critical role in tumor cell resistance to TRAIL (103, 108). Furthermore, downregulation of proapoptotic proteins, in particular Bax, accompanied by suppression of DR4/5 expression and also activation contributes to tumor-cell resistance to TRAIL (109–111). Recent findings have delivered proof of the theory that human MSCs engineered to produce and deliver TRAIL can efficiently infiltrate to and eradicate tumor cells *in vitro* and *in vivo* (112–114). For instance, Mueller et al. found that MSC with lentiviral TRAIL expression (MSC-TRAIL) abrogated the proliferation of TRAIL-resistant colorectal carcinoma (CRC) cells in a murine model possibly mediated by prolonged exposure to TRAIL (115).

### TRAIL Delivery by MSCs

The recent finding has shown that MSC-based delivery of TRAIL can target and eliminate CD133+ non-small-cell lung carcinoma (NSCLC)-derived cancer stem cells (CSCs) by modifying mitochondria membrane potential, and subsequently triggering intrinsic apoptosis in CSCs (116). Moreover, TRAIL-secreting MSCs induced robust apoptosis in lung A549, breast MDAMB231, squamous H357, and cervical Hela cancer cells in coculture experiments, and also in xenografts (117). Injected MSC-TRAIL could induce significant attenuation in metastatic tumor volume with frequent elimination of metastases in tumor xenografts (117). Importantly, MSC-TRAIL induced apoptosis in neuroblastoma cell lines *in vitro*, infiltrated tumor sites *in vivo*, and abrogated neuroblastoma development in xenotransplantation experiments following intraperitoneal injection (118). Additionally, TRAIL-secreting BMMSCs triggered apoptosis in heat-shock-treated liver cancer cells as evidenced by upregulated caspase-3 activation, and also suppressed tumor growth in tumor xenografts leading to prolonged mice survival (119). Similarly, UCMSC-TRAIL stimulated apoptosis in myeloma U-266 cells *in vitro*, and also in SCID mice models through caspase-3 activation (120). On the other hand, it was found that combine treatment of MSC-TRAIL and paclitaxel (121) or with AKT inhibitors (122) or with VPA (52) triggered apoptosis in human pancreatic carcinoma (CFPAC-1) (54), glioblastoma (U87-MG) (121), prostate cancer (PC3, LNCaP, and C4-2B) (122), and in glioblastoma (U87 and U138) (52) cell lines *in vitro*, respectively.

In sum, engineered MSCs to overexpress TRAIL have resulted in promising consequences in tumor xenografts by triggering apoptosis intrinsic and extrinsic pathways.

A summary of preclinical studies respecting TRAIL delivery using MSCs is listed in Table 4.

**Table 4:** The overview of studies based on the use of mesenchymal stem/stromal cells (MSCs) as a carrier for delivery of TRAIL to treat human tumors (*in vitro* and *in vivo*).

**Cancer**	**Cell line/model**	**Result (Ref)**
Neuroblastoma	Tumor-bearing NOD/SCID mice	MSC-TRAIL migration to tumor tissue resulted in abrogated tumor growth in xenografts (118)
NSCLC	H460 and H2170 cell line	Inducing the apoptosis intrinsic pathway by affecting mitochondria membrane potential and also NFKB1, BAG3, MCL1, GADD45A, and HRK expression (116)
Breast cancer	MCF-7 cell line	Induced apoptosis of MCF-7 cells co-cultured with modified MSC-coexpressing Smac and TRAIL (123)
SCC	H357 cell line	Induction of apoptosis of tumor cells along with suppressing colony formation (124)
NSCLC	A549 cell line	
Various cancers	A549, MDAMB23, H357, and Hela cell line	Inducing all cell lines apoptosis *in vitro* (117)
	Tumor-bearing NOD/SCID mice	Abrogation of tumor growth in subcutaneous xenograft (117)
Esophageal cancer	Eca-109 cell line	Inhibition of the proliferation and induction of apoptosis in Eca-109 cells (125)
	Eca-109 cell-bearing BALB/c nude mice	Suppression of tumor growth in xenografts (125)
Multiple myeloma	U-266 cell line	Inducing apoptosis in U-266 cells *in vitro* (120)
	U-266 cell-bearing SCID mice	Attenuation of tumor burden by selective stimulation of apoptosis in U-266 cells stimulated by caspase-3 activation *in vivo* (120)
NSCLC	A549 cell-bearing mice	Marked regression in tumor growth in xenografts (126, 127)
Pancreatic cancer	CFPAC-1 cell line	Enhancement of the antitumor effects the of MSC-TRAIL secretome by priming with paclitaxel *in vitro* (121)
Glioblastoma	U87-MG cell line	
HCC	MHCC97-H cell line	Induction of apoptosis in MHCC97-H cells co-cultured with cisplatin plus MSC-TRAIL by upregulation of death receptor 5 (DR5) *in vitro* (128)
	Tumor cell-bearing BALB/c nude mice	Abrogation of tumor growth in MHCC97-H xenografts by combination therapy using cisplatin plus MSC-TRAIL (128)
HCC	N1-S1, HepG2, and MHCC97-H cell line	Inducing apoptosis in tumor cells by upregulation of caspase-3, and DR4 and DR5 expression (119)
	HS-N1-S1 cell-bearing nude mice	Inhibition of tumor growth leading to improved survival (119)
Melanoma	B16F0 cell-bearing nude mice	Suppression of tumor growth and reduction of tumor weights (129)
Brain metastatic breast cancer	MDA-MB-23-bearing SCID mice	Induction of selective apoptosis in tumor cells by MSCs modified to co-overexpress CXCR4 and TRAIL (130)
SCC	Tumor cell-bearing nude mice	Marked inhibition in tumor growth *in vivo* (131)
Glioma	U-87MG cell-bearing nude mice	Enhancing the MSC-TRAIL tumor tropism and subsequent tumor counteraction by irradiation in glioma xenografts (132)
Mesothelioma	Isoflurane-induced NOD/SCID mice	Efficient homing of the MSC-TRAIL to malignant pleural mesothelioma and reducing the tumor growth (133, 134)
	HMESO cell-bearing SCID mice	
Glioma	U87MG cell xenografts	Significant and selective elimination of malignant cells supporting prolonged survival in xenografts (135)
Colon cancer	HCT116 cell-bearing CD1 nude mice	Induction of the p53-independent antitumor effects by combine treatment of MSC-TRAIL and 5-fluorouracil (136)
Ewing sarcoma	A-673, SK-N-MC, and SK-ES-1 cell line	Stimulating apoptosis by cell-to-cell contact in all cell lines (137)
	A-673 cell-bearing nude mice	Suppressed tumor growth in xenografts by inducing the caspase activation (137)

*TRAIL/Apo2L, tumor necrosis factor (TNF)-related apoptosis-inducing ligand; NSCLC, nonsmall-cell lung carcinoma; SCC, squamous cell carcinoma; HCC, hepatocellular carcinoma; BAG3, BAG cochaperone 3; MCL1, myeloid cell leukemia 1; GADD45A, growth arrest and DNA damage-inducible alpha; HRK, Harakiri*.

## Conclusion and Future Prospect

The MSC-based gene delivery is recently introduced as an encouraging therapeutic approach to tumor therapy, including solid tumors and hematological malignancies (138). The modified MSCs can robustly and specifically affect transformed cells without significant unwanted effects and also systemic toxicity. The strong tumor tropism of MSCs makes them reliable candidates as gene delivery vehicles, providing sustained and continued releases of antitumor cytokine. Based on the recent reports, MSCs can unfavorably support tumor progress by a diversity of mechanisms, containing the stimulation of drug resistance, proangiogenic functions, and eliciting metastasis procedure by stimulation of epithelial-mesenchymal transition (EMT) and also enrichments of the cancer stem cell (CSC) niche (139, 140). MSC-derived factors are reliable for the listed unwanted effects, affecting the various hallmarks of cancer. Nonetheless, homing potential of MSCs introduces them as a reliable option for cytokines and other antitumor drug delivery. More comprehensive investigations concerning the tumor-supportive mechanisms of MSCs can ameliorate the possibility to use them to treat cancers by optimizing their expansion, and thereby attenuation of the tumor cell growth. Besides, further knowledge of the specific molecular mechanisms complicated in the protumorigenic activities of MSCs is urgently required. Importantly, an alternative plan for using the intact MSCs for cytokine delivery is the utilizing MSC-derived conditioned medium, which potently attenuates the cell growth of MSC-derived tumor cell (47, 141, 142).

Overall, we deduce that deterioration of the MSC tumor-supportive competencies using several methods, in particular, combines treatment with engineered MSCs and small molecules (e.g., tyrosine kinase inhibitors) can result in a remarkable safety concurrently more desired therapeutic efficacy.

## Author Contributions

ER, RM, FM, SS, DB, and WA drafted the main text, figures, and tables. MJ and FT supervised the work and provided comments and additional scientific information. SC, RM, and ER reviewed and revised the text. All authors contributed to the conception and the main idea of the work and read and approved the final version of the work to be published.

## Conflict of Interest

The authors declare that the research was conducted in the absence of any commercial or financial relationships that could be construed as a potential conflict of interest.

## Publisher's Note

All claims expressed in this article are solely those of the authors and do not necessarily represent those of their affiliated organizations, or those of the publisher, the editors and the reviewers. Any product that may be evaluated in this article, or claim that may be made by its manufacturer, is not guaranteed or endorsed by the publisher.
